The article "MiR-31 promotes Th22 differentiation through targeting Bach2 in coronary heart disease" was published in 2019. Journal: Biosci Rep.

# MiR-31 promotes Th22 differentiation through targeting Bach2 in coronary heart disease

**DOI:** 10.1042/BSR20190986

**Published:** 2019-09-20

**Authors:** Rimao Huang, Xuliang Chen, Yadong Long, Ri Chen

**Affiliations:** Department of Cardiovascular Surgery, Xiangya Hospital of Centre-south University, No.87 Xiangya Road, Kaifu District, Changsha 410008, Hunan, China

**Keywords:** Bach2, CHD, miR-31, Th22 differentiation

## Abstract

The aim of the present study was to investigate the role of miR-31 in Th22 differentiation in coronary heart disease (CHD). Th22 frequencies in peripheral blood of CHD patients and controls as well as in CD4^+^ T cells were detected by flow cytometry. The mRNA expression of Th22-associated transcription factor aryl hydrocarbon receptor (AHR) and Th22-effector cytokine interleukin (IL)-22, as well as miR-31 were examined by quantitative real-time PCR (qRT-PCR). The protein level of BTB domain and CNC homolog 2 (Bach2) was measured by Western blotting. The interaction between miR-31 and Bach2 was verified using dual luciferase reporter assay. The results showed that Th22 frequency and miR-31 expression were elevated in CHD patients. Furthermore, miR-31 mimic and Bach2 silencing significantly promoted Th22 frequency and the levels of AHR and IL-22 in CD4^+^ T cells from CHD patients. Further studies showed that miR-31 facilitated Th22 cell differentiation by targeting and inhibiting Bach2. Our data indicate that miR-31 promotes Th22 differentiation through targeting Bach2 in CHD.

## Introduction

Coronary heart disease (CHD) is a growing public health problem and a leading cause of morbidity and mortality in modern society [1], which usually results from atherosclerosis [2]. Atherosclerosis is a complex chronic inflammatory disease characterized by a persistent inflammation of the arterial wall [3]. At present, although invasive coronary angiography is the gold standard for the diagnosis of CHD, there still are limitations for CHD treatment due to its invasiveness and related complications. Hence, there is an acute need for searching objective and non-invasive diagnostic biomarkers in CHD.

T cells are present during all stages of atherosclerosis suggesting that they are essential in the initiation as well as the progression of plaque [4]. Previous studies suggested that a variety of immune cell types are involved in CHD and atherosclerosis, including Treg, Th17, Th1, and Th2 cells [5–7]. Th22 cells, newly discovered Th cells that produce interleukin (IL)-12, have been recognized as the major players in inflammatory and autoimmune diseases [8–10]. Coronary plaque rupture resulted from multiple factors can lead to thrombosis and format acute coronary syndrome. Zhang et al. [11] revealed that Th22 cells and IL-22 level were significantly increased in acute myocardial infarction and unstable angina patients when compared with stable angina patients and healthy controls. Lin et al. [12] observed a significant increase in the peripheral Th22 number, IL-22 level, and aryl hydrocarbon receptor (AHR) expression in patients with acute coronary syndrome compared with those in the control group. AHR is a key specific transcription factor of Th22 cells. These above-mentioned findings suggest that there is a close link between Th22 and CHD pathogenesis.

The article "MiR-31 promotes Th22 differentiation through targeting Bach2 in coronary heart disease" was published in 2019. Journal: Biosci Rep.

MicroRNAs (miRNAs) are small (∼21 nucleotides) endogenously expressed RNAs that negatively regulate gene expression. MiRNAs play an essential role in regulating diverse biological processes including cell apoptosis, differentiation, proliferation, and metabolism [13]. Emerging evidence suggests that several miRNAs act as key regulators in the development of cardiovascular diseases [14–17]. Some miRNAs have been shown to be widely dysregulated in IL-22-producing T cells [18]. Maximilian and others [19] performed whole-genome microarray analysis and compared mRNA expression profiles of naïve CD4^+^ T cells to sort Th17 cells and Th22 cells. They found that miR-31 was up-regulated in Th22 cells and showed a positive correlation with IL-22 production [19].

BTB domain and CNC homolog 2 (Bach2) has been identified as a critical regulator in the CD4^+^ T-cell differentiation that prevents inflammatory disease by controlling the balance between tolerance and immunity. Bach2 was required for stabilizing the Treg-mediated immune homeostasis through repressing the differentiation programs of multiple effector lineages in CD4^+^ T cells [20]. Accumulating evidence has shown that Bach2 plays important roles in the differentiation of Th1, Th2, and Th17 cells by inhibiting the expression of T-lymphocyte transcription factors such as GATA3 and IRF4 [21–23]. Bach2-deficient T cells show spontaneous activation and produce high levels of Th1/Th2-type cytokines. Without Bach2, Treg cells exhibit decreased Foxp3 expression, resulting in severe chronic inflammation [24]. To the best of our knowledge, little is known about the role of Bach2 in Th22 cells.

Our bioinformatics analysis revealed that Bach2 might act a target of miR-31. Thus, in the current study, we hypothesized that miR-31 promoted AHR expression and promoted Th22 cell differentiation and IL-22 expression by targeting Bach2 in the context of CHD.

## Materials and methods

### Study population

A total of 103 individuals (61 males and 42 females, mean age 59.2 years) who underwent coronary angiography for suspected or known coronary atherosclerosis at the Xiangya Hospital of Centre-south University were enrolled in the present study. Among them, 56 CHD patients (34 males and 22 females, age 39–77 years) and 47 non-CHD subjects (27 males and 20 females, age 37–73 years) with angiographic exclusion of CHD served as the control group. The following exclusion criteria were used: infectious processes within 2 weeks, previous myocardial infarction within 6 months, spastic angina pectoris, adrenal dysfunction, thyroid dysfunction, previous revascularization procedures, neoplastic disease, advanced liver disease, autoimmune disease, and severe heart failure (NYHA classes III–IV). Clinical characteristics between two groups were shown in Table 1. The present study was approved by the human ethics committee of Xiangya Hospital of Centre-south University, and written informed consent was obtained from all participants.

The article "MiR-31 promotes Th22 differentiation through targeting Bach2 in coronary heart disease" was published in 2019. Journal: Biosci Rep.

**Table 1:** Comparison of clinical characteristics between two groups

	Non-CHD (*n*=47)	CHD (*n*=56)
Age	48 ± 12.1	50 ± 11.5
BMI (kg/m^2^)	22.12 ± 1.54	25.13 ± 2.47*
TC (mmol/l)	4.25 ± 0.88	5.04 ± 0.72*
TG (mmol/l)	1.68 ± 0.84	1.75 ± 0.91
LDL-C (mmol/l)	2.14 ± 0.75	2.78 ± 1.01*
HDL-C (mmol/l)	1.20 ± 0.25	1.25 ± 0.31
Hs-CRP (mg/l)	3.21 ± 0.64	5.05 ± 1.15*

* *P*<0.05 vs. non-CHD.

### Cell transfection and cell treatments

Peripheral whole blood samples were collected from CHD patients and non-CHD subjects and preserved with heparin. Peripheral blood mononuclear cells (PBMCs) were freshly isolated by density gradient centrifugation. CD4^+^ T cells were then purified from PBMCs by magnetic-activated cell sorting (Miltenyi, Bergisch Gladbach, Germany), and cultured in human T-cell culture medium (Lonza, Walkersville, MD, U.S.A.). Then CD4^+^ T cells were transfected with negative control, miR-31 mimic or inhibitor, si-Bach2, lentiviruses vector overexpressing Bach2 (Lv-Bach2) using T cell Nucleofector Kits according to the manufacturer’s instructions. Forty-eight hours after transfection, cells were collected for further analysis.

Th22 differentiation was subsequently induced after transfection by culturing cells in differentiation medium (growth medium supplemented with 10 ng/ml IL-1β, 30 ng/ml IL-6, 20 ng/ml IL-23, 400 nM FICZ, and 10 μM TGF-β receptor inhibitor Galunisertib).

### ELISA

The supernatant from peripheral whole blood samples was measured with IL-22 ELISA kits (Abcam, Cambridge, MA, U.S.A.) according to the manufacturer’s instructions. The concentration was calculated according to the corresponding value of optical density (OD).

### Western blotting

Total proteins were extracted from CD4^+^ T cells using RIPA lysis buffer (Beyotime, Shanghai, China) and quantified with the BCA kit (Beyotime). Equal volume of proteins were subjected to SDS/PAGE and transferred on to PVDF membrane. After blocking in PBS with 5% non-fat milk and 0.05% Tween-20 for 1 h at room temperature, the membrane was incubated overnight at 4°C with corresponding primary antibody of Bach2 (1:500; Abcam), followed by incubation for 2 h with secondary antibodies conjugated with horseradish peroxidase at room temperature. The ECL kit was used to detect immunoreactive bands according to the manufacturer’s instructions (Thermo Scientific, Waltham, MA, U.S.A.).

The article "MiR-31 promotes Th22 differentiation through targeting Bach2 in coronary heart disease" was published in 2019. Journal: Biosci Rep.

### Flow cytometric analysis

Heparinized peripheral whole blood (400 ml) in an equal volume of Roswell Park Memorial Institute (RPMI) 1640 medium were incubated for 4 h at 37°C with 5% CO_2_ in the presence of phorbol myristate acetate (PMA, 25 ng/ml, Sigma), ionomycin (1 μg/ml, Sigma), and monensin (1.7 μg/ml, BD GolgiStop). PMA and ionomycin are pharmacological T-cell activating agents. Monensin was used to block intracellular transport mechanisms, thereby leading to an accumulation of cytokines in the cells. After incubation, the cells were stained with PE-Cy5-conjugated anti-CD4 monoclonal antibodies (clone: RPA-T4, BD Biosciences, San Jose, CA) at room temperature in the dark for 20 min to delimitate CD4^+^ T cells. After staining, the cells were fixed and permeabilized. Then the cells were stained with FITC-conjugated anti-interferon (IFN)-γ monoclonal antibodies (clone: 4S-BS; 1:100; eBioscience, San Diego, CA, U.S.A.), PE–conjugated anti-IL-17A monoclonal antibodies (clone: eBio64DEC17; 1:100; eBioscience) and APC–conjugated anti-IL-22 monoclonal antibodies (clone: 22URTI; 1:100; eBioscience). Stained cells were analyzed by flow cytometric analysis using a FACS cytometer (BD Bioscience) and data were analyzed using FlowJo software (Tree Star Inc. San Carlos, CA, U.S.A.). Th22 cells were defined as CD4^+^IFN-γ-IL-17-IL-22^+^ T cells. Briefly, lymphocytes were gated by forward and side scatter and then were analyzed for IFN-γ producing and CD4 expression T cells. CD4^+^ IFN-γ cells were gated in upper left quadrant (red frame) and analyzed for IL-17 and IL-22 producing T cells. Numbers represent the percentage of cells in the quadrants. The percentages of circulating Th22 cells (Q1, % of CD4^+^IFN-γ cells) were shown.

### Quantitative real-time PCR

IL-22, AHR, and Bach2 expression in CD4^+^ T cells were measured by quantitative real-time PCR (qRT-PCR). Total RNA was extracted from cells using TRIzol reagent (Invitrogen, Carlsbad, CA, U.S.A.) according to the manufacturer’s instructions. The RNA was transcribed into first-strand complementary DNA (cDNA) using a qPCR cDNA kit (Toyobo, Osaka, Japan), and the transcripts were quantified using the SYBR Premix ExTaq™ II reagent (Takara, Japan) and a Lightcycler 480 Real-time PCR System (Roche). The mRNA levels of IL-22, AHR, and Bach2 were normalized to that of GAPDH. MiRNA in CD4^+^ T cells was extracted using the miRVana extraction kit (Ambion, Austin, TX). For quantification, miRNA qRT-PCR Primer Set (Ribo Life Science Co. Ltd., China) and M-MLV Reverse Transcriptase (Takara Biotechnology, China) were used for measuring miR-31 expression. U6 was used as the internal control for miR-31. All data were analyzed using LightCycler 480 Real-time Analysis Sofware.

The article "MiR-31 promotes Th22 differentiation through targeting Bach2 in coronary heart disease" was published in 2019. Journal: Biosci Rep.

### Dual luciferase reporter assay

The 3′-UTR of Bach2 was amplified from human cDNA. The wild-type fragment containing the predicted miR-31 binding site and its mutant fragment were obtained from 3′-UTR of Bach2. Amplicons were inserted between SacI and XbaI cleavage sites of pmirGLO vector (Promega, U.S.A.). The human embryonic kidney cell line (HEK293T) was selected on the basis of the low endogenous miRNA expression. Cells were seeded in 24-well plates. When it reached 70–80% confluence, the 800 ng wild-type or mutant reporter and 20 μM miR-31 mimic, inhibitor (GenePharma Co., Ltd, China) were co-transfected into HEK293T cells using Lipofectamine 2000 (Invitrogen, U.S.A.). Twenty-four hours after transfection, firefly and *Renilla* luciferase activities were measured in cell lysates using the dual-luciferase reporter system.

### Statistical analysis

All data were analyzed with SPSS 16.0. Data were presented as mean ± standard deviation (SD). Student’s *t* test was used to analyze differences between two groups. One-way ANOVA analysis was used to analyze differences among multiple groups. Differences at *P*< 0.05 were considered to be statistically significant.

## Results

### Th22 frequency and miR-31 expression are elevated in CHD patients

To assess whether Th22 cells were involved in the development of CHD, we initially examined the frequency of Th22 cells in peripheral blood from CHD patients and non-CHD subjects by flow cytometry. Representative flow cytometry results and quantitative results showed that the frequency of Th22 cells was notably increased in peripheral blood from CHD patients compared with non-CHD participants (Figure 1A). ELISA results showed that the level of IL-22 in peripheral blood was significantly elevated in CHD group compared with non-CHD group (Figure 1B). To explore the correlation between Th22 cells count and miR-31 expression in CHD patients, we also measured the mRNA level of miR-31 in peripheral blood. The results of qRT-PCR demonstrated that miR-31 expression in peripheral blood was higher in the CHD group when compared with the non-CHD group (Figure 1C). In addition, we isolated CD4^+^ IFN-γ-IL-17-IL-22^+^ (Th22) cells from subjects and then examined expression of IL-22 and miR-31 by qRT-PCR. Consistent with data in peripheral blood, IL-22 mRNA expression (Figure 1D) and miR-31 expression (Figure 1E) in Th22 cells were notably higher in the CHD group when compared with the non-CHD group.

The article "MiR-31 promotes Th22 differentiation through targeting Bach2 in coronary heart disease" was published in 2019. Journal: Biosci Rep.

**Figure 1:** Th22 frequency and miR-31 expression were elevated in CHD patients (**A**) Representative flow cytometry results of Th22 frequency in peripheral blood of CHD patients and non-CHD subjects. (**B**) ELISA results of IL-22 in peripheral blood of CHD patients and non-CHD subjects. (**C**) QRT-PCR results of miR-31 in peripheral blood of CHD patients and non-CHD subjects. (**D,E**) QRT-PCR results of IL-22 (D) and miR-31 (E) in CD4^+^ IFN-γ-IL-17-IL-22^+^ (Th22) cells from CHD patients and non-CHD subjects. *n*=56 in CHD group and *n*=47 in non-CHD group. *P<0.05 vs. non-CHD. Abbreviation: non-CHD, angiographic exclusion of CHD.

### MiR-31 facilitates Th22 cell differentiation

To study the role of miR-31 in Th22 cell differentiation, we transfected miR-31 mimic, inhibitor, or their controls into isolated CD4^+^ T cells from patients. Flow cytometry results showed miR-31 mimic significantly promoted Th22 differentiation in CD4^+^ T cells compared with mimic control while miR-31 inhibitor prominently repressed Th22 differentiation compared with inhibitor control (Figure 2A). Concordantly, miR-31 mimic facilitated the expression of Th22-associated transcription factor AHR in CD4^+^ T cells relative to mimic control while miR-31 inhibitor prominently repressed AHR expression relative to inhibitor control (Figure 2B). qRT-PCR and ELISA results showed a similar pattern that miR-31 mimic significantly increased IL-22 secretion in CD4^+^ T cells (Figure 2C,D). Given that, miR-31 facilitates Th22 cell differentiation.

**Figure 2:** MiR-31 facilitates Th22 cell differentiation CD4^+^ T cells isolated from peripheral blood were transfected miR-31 mimic, mimic NC, miR-31 inhibitor or inhibitor NC. (**A**) Representative flow cytometry results of Th22 frequency in transfected CD4^+^ T cells. (**B**) Expression of Th22-associated transcription factor AHR in transfected CD4^+^ T cells was analyzed by qRT-PCR. (**C**) The mRNA expression of IL-22 in transfected CD4^+^ T cells was analyzed by qRT-PCR. (**D**) The levels of IL-22 in transfected CD4^+^ T cells supernatant was analyzed by ELISA. Data were presented as mean ± SD (*n*=3). *P<0.05 vs non-CHD; ^#^*P*<0.05 vs mimic NC; ^&^*P*<0.05 vs inhibitor NC. Abbreviations: NC, negative control; non-CHD, angiographic exclusion of CHD.

The article "MiR-31 promotes Th22 differentiation through targeting Bach2 in coronary heart disease" was published in 2019. Journal: Biosci Rep.

### Bach2 silencing facilitates Th22 cell differentiation

Next, we examined the function of Bach2 in Th22 cell differentiation. Flow cytometry results showed Bach2 silencing notably promoted Th22 differentiation in CD4^+^ T cells compared with scramble control (Figure 3A). Furthermore, Bach2 silencing significantly decreased expression of Th22-associated transcription factor AHR (Figure 3B) and secretion of IL-22 in CD4^+^ T cells (Figure 3C,D). These data indicated that Bach2 silencing facilitates Th22 cell differentiation.

**Figure 3:** Bach2 silencing facilitates Th22 cell differentiation CD4^+^ T cells isolated from peripheral blood were transfected as si-Bach2 or scramble siRNA control (si-NC). (**A**) Representative flow cytometry results of Th22 frequency in transfected CD4^+^ T cells. (**B**) Expression of Th22-associated transcription factor AHR in transfected CD4^+^ T cells was analyzed by qRT-PCR. (**C**) The mRNA expression of IL-22 in transfected CD4^+^ T cells was analyzed by qRT-PCR. (**D**) The levels of IL-22 in transfected CD4^+^ T cells supernatant was analyzed by ELISA. Data were presented as mean ±SD (*n*=3). *P<0.05 vs non-CHD; ^#^*P*<0.05 vs si-NC. Abbreviations: NC, negative control; non-CHD, angiographic exclusion of CHD.

### MiR-31 facilitates Th22 cell differentiation by targeting Bach2

To gain insight into the underlying mechanisms, miRNA target gene prediction site TargetScan was used to predict potential targets of miR-31. Among the candidates, we found a highly conservative and specific combination sequence between miR-31 and Bach2 3′-UTR (Figure 4C). Results of qRT-PCR showed that miR-31 expression was higher (Figure 4A), whereas Bach2 mRNA expression was lower (Figure 4B) in Th22^+^CD4^+^ T cells from CHD patients when compared with the Th22^+^CD4^+^ T cells group. Furthermore, miR-31 mimic significantly repressed luciferase activity when co-transfected with reporter containing WT Bach2 3′UTR but not MUT Bach2 3′UTR (Figure 4C). The mimic and inhibitor of miR-31 were transfected into CD4^+^ T cells to examine the effect of miR-31 on Bach2 expression. Compared with controls, miR-31 overexpression significantly suppressed Bach2 expression, while miR-31 inhibitor induced Bach2 expression in CD4^+^ T cells from CHD patients, both at mRNA and protein levels (Figure 4D). These data indicated that miR-31 targets and inhibits Bach2 expression.

**Figure 4:** MiR-31 targets and inhibits Bach2 expression (**A,B**) qRT-PCR results of miR-31 (A) and IL-22 (B) in Th22^−^CD4^+^ T cells and Th22^+^CD4^+^ T cells from CHD patients. (**C**) Schematic of the putative miR-31 target site in human Bach2 3′-UTR and the seven mutated nucleotides are colored red. Luciferase report assay delineated a reduction in luciferase activity of Bach2-WT reporter after introduction of miR-31 in HEK293T cells. (**D**) qRT-PCR and Western blotting analysis of Bach2 in CD4^+^ T cells transfected with miR-31 mimic, miR-31 inhibitor, and corresponding controls. Data were presented as mean ± SD (*n*=3). *P<0.05 vs Th22^−^CD4^+^ T cells or non-CHD; ^#^*P*<0.05 vs mimic NC; ^&^*P*<0.05 vs inhibitor NC.

The article "MiR-31 promotes Th22 differentiation through targeting Bach2 in coronary heart disease" was published in 2019. Journal: Biosci Rep.

Finally, we performed rescue experiments to elucidate whether miR-31 facilitated Th22 differentiation through inhibiting Bach2 expression. To this end, naive CD4^+^ T cells were transfected with miR-31 mimic or Lv-Bach2, followed by stimulation with 10 ng/ml IL-1β, 30 ng/ml IL-6, 20 ng/ml IL-23, 400 nM FICZ, and 10 μM TGF-β receptor inhibitor Galunisertib to activate naive CD4^+^ T cells to differentiate into Th22 cells. As shown in Figure 5A, low-level expression of Bach2 was detected in treated cells in the presence of miR-31 mimic, but the decreased Bach2 expression was restored by Bach2 overexpression. More importantly, Bach2 overexpression in induced CD4^+^ T cells effectively impaired the ability of miR-31 mimic to increase Th22 frequency (Figure 5B). Furthermore, the levels of AHR and IL-22 in induced CD4^+^ T cells were markedly down-regulated when the cells were co-transfected with Lv-Bach2 and miR-31 mimic compared with the miR-31 mimic group (Figure 5C–E). Together, these data indicated that Bach2 overexpression significantly abrogated the miR-31 mimic-mediated promotion of Th22 differentiation. Thus, our data indicated that miR-31 facilitates Th22 cell differentiation, at least in part, by targeting and inhibiting Bach2.

**Figure 5:** MiR-31 facilitates Th22 cell differentiation by targeting Bach2 Naive CD4^+^ T cells were transfected with miR-31 mimic or Lv-Bach2, Th22 differentiation was induced by 10 ng/ml IL-1β, 30 ng/ml IL-6, 20 ng/ml IL-23, 400 nM FICZ and 10 μM TGF-β receptor inhibitor Galunisertib. (**A**) Bach2 expression in CD4^+^ T cells was determined by qRT-PCR and Western blotting. (**B**) Th22 frequency in CD4^+^ T cells was determined by flow cytometry. (**C,D**) The expressions of AHR (C) and IL-22 (D) in CD4^+^ T cells were analyzed by qRT-PCR. (**E**) IL-22 level in CD4^+^ T cells was analyzed by ELISA. Data were presented as mean ± SD (*n*=3). *P<0.05 vs control; ^#^*P*<0.05 vs mimic NC+Th22 culture; ^&^*P*<0.05 vs mimic NC+Lv-NC+Th22 culture.

## Discussion

In the present study, increased Th22 frequency and miR-31 expression were observed in patients with CHD. Moreover, miR-31 elevated the Th22 cell proportion and Th22-related cytokine secretion in CHD patients. Furthermore, we found that miR-31 facilitated Th22 cell differentiation by targeting and inhibiting Bach2. Our findings add a new clue to the regulation of Th22 differentiation by miRNAs in CHD.

The article "MiR-31 promotes Th22 differentiation through targeting Bach2 in coronary heart disease" was published in 2019. Journal: Biosci Rep.

Researches have demonstrated that Th22 cells, by producing pro-inflammatory cytokines such as IL-22, were implicated in the pathogenesis of various inflammatory diseases and autoimmune diseases [9]. For instance, elevated numbers of Th22 cells were observed in peripheral blood of patients with psoriasis, suggesting that Th22 cells may contribute to cutaneous inflammation and systemic inflammatory disease [25]. Besides, Th22 cells and IL-22 level were significantly elevated in patients with rheumatoid arthritis (RA) and ankylosing spondylitis (AS) when compared with healthy controls, indicating that Th22 cells may be implicated in the pathogenesis of AS and RA [26,27]. The present study also revealed an increased level of Th22 cells in patients with CHD.

Zhang et al. [11] revealed that Th22 cells and IL-22 level were significantly increased in unstable angina patients when compared with stable angina patients and healthy controls. Lin et al. [12] observed a significant increase in the peripheral Th22 number, AHR expression, and IL-22 level in patients with acute coronary syndrome compared with those in the control group. In addition, elevated serum IL-22 was independently correlated with the incidence of CHD. Conversely, it has been shown that IL-22 protects endothelial cells from glucose- and lysophosphatidylcholine-induced injury [28]. Furthermore, Fatkhullina et al. [29] reported that IL-22 restricted atherosclerosis by repressing pro-atherogenic microbiota. They found that ablation of IL-22 exacerbates atherosclerosis and IL-22 administration suppresses the atherosclerosis development [29]. Coronary artery atherosclerosis is the leading cause of CHD [30]. Thus, these above-mentioned findings suggest that Th22 cells may participate in the pathogenesis of CHD by IL-22 secretion [31]. Our results showed that miR-31 promotes Th22 differentiation through targeting Bach2 in CHD, indicating that miR-31 might play a role in the pathogenesis of CHD. However, the exact role of miR-31-Bach2-Th22-IL-22 pathway involved in CHD needs to be further studied.

MiRNAs are increasingly recognized as important modulators in regulating the motility and plasticity of lymphocytes through interfering with related-signal transduction pathways [32,33]. miRNAs might be responsible for the persistence of pro-inflammatory Th1 cells in the inflamed tissues, by inhibiting several genes involved in related signaling pathways [34]. Mounting studies have described biological role of miR-31 in a wide range of diseases [35,36]. It has been shown that miR-31 recedes the activity of pro-inflammatory Th1 cells through regulating the expression of genes which are involved in the rearrangement of actin cytoskeleton downstream of TCR signaling [37]. Our work showed up-regulated miR-31 and IL-22 expression in patients with CHD. Further study demonstrated that miR-31 facilitated the expression of AHR and IL-22 as well as frequency of Th22 in CD4^+^ T cells from CHD patients. Furthermore, we identified miR-31 directly targeted and inhibited Bach2 expression in CD4^+^ T cells. Bach2 is weakly expressed in CD4^+^ T cells from patients with CHD, and miR-31 mimic significantly suppressed Bach2 expression. Moreover, the effect of miR-31 mimic on Th22 frequency and the levels of AHR and IL-22 in CD4^+^ T cells were markedly reversed by Bach2 overexpression, indicating that miR-31 facilitates Th22 cell differentiation by targeting Bach2.

The article "MiR-31 promotes Th22 differentiation through targeting Bach2 in coronary heart disease" was published in 2019. Journal: Biosci Rep.

In summary, our findings demonstrate that miR-31 facilitates Th22 cell differentiation by targeting Bach2 expression in the setting of CHD. These data indicated that regulation of Th22 cell differentiation by miR-31 might play a role in the pathogenesis of CHD.

## Abbreviations

AHR: aryl hydrocarbon receptor
APC: allophycocyanin
AS: ankylosing spondylitis
Bach2: BTB domain and CNC homolog 2
cDNA: complementary DNA
CHD: coronary heart disease
GATA3: GATA binding protein 3
IFN: interferon
IL: interleukin
Lv-Bach2: lentivirus vector overexpressing Bach2
miRNA: microRNA
NYHA: the New York Heart Association
PBMC: peripheral blood mononuclear cell
PE: phycoerythrin
PMA: phorbol myristate acetate
qRT-PCR: quantitative real-time PCR
RA: rheumatoid arthritis
RIPA: radio-immunoprecipitation assay
TCR: T cell receptor
Th: T helper
Treg: T regulatory
